# Upregulated Tripartite Motif 47 Could Facilitate Glioma Cell Proliferation and Metastasis as a Tumorigenesis Promoter

**DOI:** 10.1155/2021/5594973

**Published:** 2021-03-25

**Authors:** Bin Ji, Lijuan Liu, Yongping Guo, Feng Ming, Jun Jiang, Fangfang Li, Guo'an Zhao, Jianyong Wen, Ning Li

**Affiliations:** ^1^Department of Neurosurgery, Changzhi People's Hospital, No. 502, Changxing Middle Road, Changzhi, Shanxi, China; ^2^Department of Blood Transfusion, Heping Hospital Affiliated to Changzhi Medical College, China; ^3^State Key Laboratory of Genetic Engineering, School of Life Sciences, Fudan University, Shanghai 200438, China

## Abstract

**Introduction:**

Tripartite motif 47 (TRIM47) belongs to a category of the TRIM family. It takes part in cancer tumorigenesis, thus demonstrating important functions across numerous carcinomas. Unfortunately, it is still elusive towards TRIM47 expression, characteristic, and biological function in brain gliomas.

**Methods:**

Public database analysis was applied to analyze TRIM47 expression, and quantitative real-time PCR (qRT-PCR) was applied to detect the expression of TRIM47 in 9 paired tissues of glioma. The Cancer Genome Atlas (TCGA) and the Chinese Glioma Genome Atlas (CGGA) databases were applied to evaluate the overall survival (OS). Gene Ontology (GO) term and Kyoto Encyclopedia of Genes and Genomes (KEGG) pathways were applied to analyze differentially expressed gene (DEG) functions. *In vitro* experiments were performed to validate TRIM47-mediated effects on glioma cell proliferation, migration, and invasion.

**Results:**

Compared to that in normal tissues, TRIM47 expression was greatly higher in glioma tissues, and its expression level was associated with different grades of glioma. Our data indicated that highly expressed TRIM47 displayed an association with the poor prognosis of glioma patients. Ablating TRIM47 obviously impeded glioma cell invasion and migration.

**Conclusion:**

TRIM47 could modulate glioma cell proliferation, invasion, and migration. Highly expressed TRIM47 exhibited a correlation with poor prognosis. All data imply that TRIM47 is a probable biomarker for glioma and has the potentiality to become a newly generated target for glioma treatment.

## 1. Introduction

Glioma is a widely occurred malignant neoplasm in the nervous system [1]. It has the characteristics of aggressiveness, immortal proliferation, no apoptosis, and no evident boundary with normal brain tissue [2]. In the light of its refractory, specific serological indicators and treatment methods are urgently essential [3]. Because of the high grade of malignancy, recurrence ratio, and morbidity, the current diagnosis of glioma primarily depends on imaging tests [4]. The treatment strategies for glioma mainly comprise surgery, radiation therapy, and chemotherapy [5]. After treatment, the 2-year survival rate in glioma patients is very low, and its prognosis is also poor [6]. Therefore, it is urgent to improve the treatment methods for glioma patients.

Tripartite motif 47 (TRIM47) protein belongs to a category of the TRIM family and participates in many cellular processes, such as cell proliferation [7]. Previous studies demonstrate that tumor tissues highly express TRIM47, compared to normal adjacent tissues [8]. Takayama et al. revealed that highly expressed TRIM47 was considered a powerful factor for prostate cancer prognosis [9]. Another study suggested that human lung carcinoma tissues and colorectal carcinoma strongly expressed TRIM47 relative to benign tissues [10, 11]. Based on what was mentioned previously, TRIM47 is a prospective biomarker for glioma and has the potentiality to become a newly generated target for glioma treatment.

In our study, we attempted to systematically validate TRIM47 function in glioma. The TRIM47 level in glioma specimens was measured, and the relationship between TRIM47 and glioma was then studied utilizing several biological assays. Our findings collectively suggested that TRIM47 could be regarded as a modulator of glioma cell development.

## 2. Materials and Methods

### 2.1. Data Processing

The levels of TRIM47 in multiple cancers and normal tissues were reviewed using Tumor Immune Estimation Resource (TIMER, https://cistrome.shinyapps.io/timer/) and Gene Expression Profiling Interactive Analysis (GEPIA, http://gepia.cancer-pku.cn/). The mRNA-seq and relevant clinical data of glioma patients were acquired from The Cancer Genome Atlas (TCGA, https://www.cancer.gov/about-nci/organization/ccg/research/structural-genomics/tcga) and the Chinese Glioma Genome Atlas (CGGA, http://www.cgga.org.cn/) database.

### 2.2. Screening Differentially Expressed Genes (DEGs)

The raw data of transcriptome profiles in highly expressed and lowly expressed TRIM47 patients were from the TCGA dataset. The R package “limma” was applied to screen the DEGs. *P* value < 0.05 and log2 fold‐change ≥ 1 were regarded as the screening thresholds for DEGs.

### 2.3. Enrichment Analysis

Gene Ontology (GO) term and Kyoto Encyclopedia of Genes and Genomes (KEGG) pathways were executed to analyze the enrichment of the DEGs. The enriched GO terms and KEGG pathway were identified by the cutoff criteria of “adjusted *P* < 0.05.”

### 2.4. Cell Culture

HEB, SW1783 (HTB-13), U373 (HTB-17), SW1088 (HTB-12), U87 (HTB-14), and A172 (CRL-1620) were from the American Type Culture Collection (Manassas, Virginia). They got maintained in DMEM with 10% FBS (Invitrogen, USA) at 37°C with 5% CO_2_.

### 2.5. Extraction and Quantitation of RNA

Whole RNA was harvested by TRIzol reagent (Invitrogen, USA). Complementary DNA (cDNA) was produced by the PrimeScript RT Kit (TaKaRa, Japan). QRT-PCR was conducted using SYBR premix Ex Taq I. GAPDH was selected as a reference. The 2^-*ΔΔ*Ct^ method was applied to tackle all the data. TRIM47 primers and GAPDH were synthesized by Sangon Biotech Co., Ltd. (Shanghai, China). Primer sequences were as follows: TRIM47, forward, 5′-CTGAGCAGTCCAAAGTCCTGA-3′; reverse, 5′-CTACGGCTGCACTCTTGATG-3′; GAPDH, forward, 5′-GGAGCGAGATCCCTCCAAAAT-3′, reverse, 5′-GGCTGTTGTCATACTTCTCATGG-3′.

### 2.6. Cell Transfection

Shanghai Gene Pharmaceutical Co., Ltd. (Shanghai, China) synthesized TRIM47 short interfering ribonucleic acid (siRNAs). si-TRIM47 and si-NC were transfected into cells by lipofectamine 2000 reagent (Invitrogen, USA). The sequences were as follows: si-TRIM47 #1, 5′-CCTCAAGTTTGCCTATATT-3′; si-TRIM47 #2, 5′-GCAGCTGTTTGGAACCAAA-3′; si-NC, 5′-UUCUCCGAACGUGUCACGUTT-3′.

### 2.7. CCK-8 Assay

Cell Counting Kit- (CCK-) 8 Assay (Dojindo Laboratories, Kumamoto City, Japan) was applied to detect cell proliferation. 5 × 10^3^ cells/well were inoculated in a 96-well plate, and 10 *μ*L of CCK-8 solution/well was supplemented at a certain time. All cells were incubated for 2 hours at 37°C incubators. The OD value of 450 nm was observed on a microplate reader (BioTek, Winooski, VT, USA). All the data were derived from three separate experiments in triplicate.

### 2.8. Transwell Assay

Transwell analysis was conducted using Transwell chambers (pore size 8 *μ*m; Costar Corporation, USA) in the presence or absence of matrigel (BD Biosciences, USA). The upper insert contained 1 × 10^5^ cells. The lower chamber included 700 *μ*L of medium with 20% FBS and was used as a chemical attractant. After 24 to 48 hours postculture, cells remaining in the lower chamber were fixed with ethanol, followed by stain using 0.2% crystal violet.

### 2.9. Kaplan-Meier Plotter Tool Analysis

The correlation between TRIM47 and glioma prognosis was assessed by the Kaplan-Meier plotter tool (http://kmplot.com/analysis/) objective. This toolset was a sort of database responsible for integrating the data of gene expression and clinical information and could be applied to analyze the prognostic value of TRIM47 in glioma.

### 2.10. Statistical Analysis

All the data were obtained from three separate experiments in triplicate one time. SPSS 17.0 software (SPSS, Inc., Chicago, IL, USA) was executed to analyze the statistics. The comparison existing in different groups was analyzed by Student's *t*-test or Mann-Whitney *U*-test as the test condition indicated. The overall survival (OS) ratio was interpreted by Kaplan-Meier. Cox proportional hazard model multivariate analysis was used to determine the TRIM47 level and clinicopathological features on OS. *P* < 0.05 with a 95% of confidence interval means an obvious difference in two or more groups.

## 3. Results

### 3.1. Evaluation of the TRIM47 Expression Level in Tumor and Adjacent Normal Tissues

GEPIA and TIMER datasets were applied to analyze the differential levels of TRIM47 in various tumor and adjacent normal tissues. The results revealed that TRIM47 was an oncogene in most tumors like cholangiocarcinoma (CHOL), esophageal carcinoma (ESCA), liver hepatocellular carcinoma (LIHC), and lung adenocarcinoma (LUAD), but it was a tumor-suppressor gene in kidney chromophobe (KICH) and prostate adenocarcinoma (PRAD). Of interest, our data suggested that the level of TRIM47 was largely raised in glioblastoma multiforme (GBM) and lower-grade glioma (LGG) tissues after GEPIA database analysis (Figure 1(a)). Nevertheless, the abovementioned regulation was not observed after TIMER database analysis (Figure 1(b)). Thus, it is necessary to make further investigation towards the relationship between TRIM47 and glioma.

### 3.2. Upregulated TRIM47 Increased Glioma Grade

Figure 2(a) which displays the level of TRIM47 was greatly associated with the WHO grade of glioma (*P* < 0.001). Heightened TRIM47 expression levels were accompanied by the increase of glioma WHO grade in the CGGA database. Additionally, after analysis of the TCGA database, the TRIM47 expression level in LGG and GBM was also significantly upregulated compared with that in normal tissues. More importantly, TRIM47 expression levels were also higher in GBM than LGG (Figure 2(b)). All the data implied that TRIM47 was a prospective oncogene in glioma and its expression was related to the grade of neoplasm.

### 3.3. The Expression Level of TRIM47 in Different Grades and Histologies of Glioma

The prognostic value of TRIM47 in glioma patients was evaluated in this part. Kaplan-Meier curve analysis was initially performed using the TCGA database. The GBM patients were composed of 81 cases of a highly expressed TRIM47 group and 81 cases of a lowly expressed TRIM47 group. Brain LGG patients were divided into 257 cases of a highly expressed TRIM47 group and 257 cases of a lowly expressed TRIM47 group. 676 cases of glioma patients contained 338 cases of a highly expressed TRIM47 group and 338 cases of a lowly expressed TRIM47 group. Figures 3(a)–3(c) suggest that highly expressed TRIM47 exhibited a significant association with shorter OS in GBM (*P* = 0.0012, Figure 3(a)), LGG (*P* = 0.042, Figure 3(b)), and glioma (*P* = 0.0017, Figure 3(c)) patients, indicating that TRIM47 might be a potential biomarker for the poor OS of glioma patient no matter in LGG or GBM. Furthermore, the CGGA database was also applied to explore the links between TRIM47 expression level and the OS of glioma patients. 111 cases of highly expressed TRIM47 and 111 cases of lowly expressed TRIM47 samples were analyzed. Our results were in line with CGGA database analysis (*P* = 0.0048, Figure 3(d)). Taken together, all these results demonstrated that high TRIM47 expression predicted poor OS and was a poor prognosis factor in glioma.

### 3.4. Identification of the Potential Biological Process and Signaling Pathways of TRIM47 Involved

Up to now, it is yet unclear about the impacts of TRIM47 on glioma proliferation and metastasis. We downloaded glioma-related data from TCGA and uploaded DEGs to the DAVID to estimate the differential GO and KEGG pathways. GO term results showed the DEGs primarily took part in the bioprocess (BP), including axonemal dynein complex, axoneme and inner dynein arm assembly, cellular response to fibroblast growth factor stimulus, inositol phosphate metabolic process, fibroblast growth factor receptor signaling pathway, assembly, miotic cell cycle phase transition, positive modulation of protein localization to chromosome telomeric region, and modulation of a p53-mediated intrinsic apoptotic signaling pathway (Figure 4(a)). KEGG pathway analysis showed that these DEGs mainly participated in cell cycle, cellular senescence, human T-cell leukemia virus 1 infection, inositol phosphate metabolism, phosphatidylinositol signaling system, signaling pathway in diabetic complications, American trypanosomiasis, glutamatergic synapse, sphingolipid and AGE-RAGE, and calcium signaling pathways (Figure 4(b)). Our data suggested that the DEGs mainly took part in the development of the nervous system extracellular matrix and the signal transduction of cell surface.

### 3.5. TRIM47 Expressed Highly in Glioma

TRIM47 expressions were determined in glioma tissues and cell lines.  Figure 5(a) reveals that compared to that in adjacent brain tissues, TRIM47 was highly expressed in 9 cases of glioma tissues. Similar results showed TRIM47 had a high expression in glioma cell lines, particularly in SW1783 (Figure 5(b)). SW1783 were therefore chosen in the following studies. For further exploring the biological functions of TRIM47 in glioma cells, we transfected siRNAs specific for TRIM47 into indicated cells as indicated. The data showed that si-TRIM47 #2 had a better knockdown effect on SW1783 (Figure 5(c)). Thus, it was selected for the next assays.

### 3.6. TRIM47 Facilitated the Cell Basic Activities in Glioma

In view of the above assays, we silenced TRIM47 in SW1783 cells by si-TRIM47 #2 to detect the impacts on cell proliferation. Our data suggested that the reduction of TRIM47 greatly hindered cell proliferation, especially in SW1783 (Figure 5(d)). SW1783 was thus selected in the following studies. Next, we further validated the impacts of TRIM47 on the migrated and invasive glioma cells. Our data suggested knocking down TRIM47 largely suppressed the cells' migrated and invasive activities (Figures 5(e) and 5(f)). In short, TRIM47 can promote the biological activities of glioma cells and tumors.

## 4. Discussion

Gliomas are the widely occurred malignant brain neoplasm [1, 12]. Amid these gliomas, the most malignant one (WHO grade IV) is glioblastoma, which is well known for its drug resistance [13]. The commonly used therapeutic strategies usually cannot obtain the expected results due to the resistance of cancer cells [14]. Herein, uncovering the mechanism of gliomagenesis and development could facilitate diagnosis and treatment of glioma in near decades [15]. Recent bioinformatic advances largely ameliorated biomedicine research, including unearthing the hub genes and verifying their respective function [16]. Herein, identifying pivotal biomarkers was conducive to improving the diagnosis and treatment of neoplasm [17].

TRIM is overexpressed in several tumors [18]. Nevertheless, it is not well understood regarding the expression, prognostic value, and function of TRIM47 in glioma [19]. In our study, TCGA and CGGA database analyses revealed that TRIM47 expression was higher in LGG or GBM than that in normal tissue. Its expression was correlated with the tumor grade. Besides, TRIM47 expression was also examined by qRT-PCR. These outcomes revealed that TRIM47 had a high expression in the samples and cell lines of glioma, not in normal tissues. All these indicated that TRIM47 might be an important indicator for gliomas and their malignancy. Thus, we further determined the potential of TRIM47 predicting the prognosis of glioma. Kaplan-Meier analysis in both TCCA and CGGA databases revealed that a higher level of TRIM47 in LGG or GBM would lead to the poor OS. Our data suggested that the level of TRIM47 could be regarded as a promising indicator for glioma prognosis.

The functions of molecules in an individual usually fulfill through interactions with others not alone only [20]. Different molecules generate a complex network of the regulation [21]. Molecules with identical expression patterns usually have a close association in function [20, 22]. TRIM47 has been reported in multiple carcinomas, but its function is not clear [23]. We thus conducted related experiments to validate the mechanism and function. We identified the DEGs in glioma patients with high and low expression of TRIM47. GO and KEGG enrichment analysis of these DEGs showed that TRIM47 might be involved in modulating cell proliferation, cell cycle, and other biological processes.

Finally, we performed the CCK-8 assay and Transwell assay to detect TRIM47 function in glioma. After knocking down TRIM47, we found that glioma cell proliferation, migration, and invasion were inhibited.

This study has limitations. The number of clinical samples is not large enough. In future studies, we will collect more clinical samples and clinical parameters of glioma patients, including age, gender, and survival time, to further explore the function of TRIM47 in glioma. In addition, the regulatory mechanism involved in TRIM47 in gliomas will be further studied.

To sum up, this study explored the role of TRIM47 in glioma for the first time. Based on public databases, we analyzed the expression level of TRIM47 in human tumors. The results showed that TRIM47 was significantly overexpressed in glioma, and the expression level of TRIM47 was positively correlated with the WHO grades of glioma. The high expression of TRIM47 had a significant correlation with the shorter OS of patients with glioma. These findings demonstrated that TRIM47 expressed highly in the glioma cells. Highly expressed TRIM47 could promote glioma cell proliferation, migration, and invasion. Our results provide a better understanding of the role in glioma. All data collectively indicate that TRIM47 is a prospective biomarker of glioma.

## Figures and Tables

**Figure 1:** Differential expression level of TRIM47 between tumors and adjacent normal tissues. (a) GEPIA database analysis of TRIM47 expression in various tumors and adjacent normal tissues. (b) TIMER database analysis of TRIM47 expression in various tumors and adjacent normal tissues (^∗^*P* < 0.05, ^∗∗^*P* < 0.01, and ^∗∗∗^*P* < 0.001).

**Figure 2:** Analysis of TRIM47 expression levels in normal tissues and glioma tissues with different grades. (a) TRIM47 expressions in different WHO grade glioma samples. (b) TRIM47 expressions in normal tissues, LGG, and GBM.

**Figure 3:** TCGA and CGGA database analyses of the correlation between TRIM47 expression and the prognosis of glioma patients. (a–c) TCGA database analysis of Kaplan-Meier curves of OS in LGG, GBM, and glioma. (d) CGGA database analysis of Kaplan-Meier curves of OS in glioma.

**Figure 4:** GO and KEGG pathway enrichment analysis of DEGs. (a) GO term analysis of top 10 biological processes of DEGs enriched. (b) KEGG pathway analysis of top 10 signaling pathways of DEGs involved.

**Figure 5:** TRIM47 highly expressed in glioma and facilitated the proliferation, migration, and invasion of glioma cells. (a) Comparison of TRIM47 in glioma tissues and normal tissues (*n* = 9) (^∗^*P* < 0.05). (b) Comparison of TRIM47 in glioma cells and normal brain cells (^∗^*P* < 0.05 and ^∗∗^*P* < 0.01). (c) Evaluation of the knockout efficiency of si-TRIM47 in SW1783 (^∗^*P* < 0.05). (d) The impacts of TRIM47 on the proliferation of glioma cells SW1783. (e, f) The impacts of TRIM47 on the invasion and migration of glioma cells SW1783 (^∗^*P* < 0.05 and ^∗∗^*P* < 0.01).

## Data Availability

The datasets used and/or analyzed during the current study are available from the corresponding author on reasonable request.
